# Diagnostic Performance of Transient Elastography Versus Two-Dimensional Shear Wave Elastography for Liver Fibrosis in Chronic Viral Hepatitis: Direct Comparison and a Meta-Analysis

**DOI:** 10.1155/2022/1960244

**Published:** 2022-09-17

**Authors:** Qing-Tian Luo, Qing Zhu, Xiao-Dan Zong, Ming-Kai Li, Hong-Sheng Yu, Chang-Yu Jiang, Xiang Liao

**Affiliations:** ^1^Department of Pain Medicine and Shenzhen Municipal Key Laboratory for Pain Medicine, Huazhong University of Science and Technology Union Shenzhen Hospital, 89 Taoyuan Ave, Nanshan District, Shenzhen, 518000. Guangdong Province, China; ^2^Guangdong Key Laboratory for Biomedical Measurements and Ultrasound Imaging, School of Biomedical Engineering, Shenzhen University Health Science Center, 1066 Xueyuan Avenue, Nanshan District, Shenzhen, 518060 Guangdong Province, China; ^3^Pain Management Department of The Second Affiliated Hospital, School of Medicine, The Chinese University of Hong Kong, Shenzhen, Guangdong, 518172, P. R. China & Longgang District People's Hospital of Shenzhen, No. 53 Aixin Road, Longcheng Street, Longgang District, Shenzhen, 518172 Guangdong Province, China; ^4^Department of Radiology, The Third Affiliated Hospital of Sun Yat-Sen University, No. 600 Tianhe Road, Guangzhou, 510000 Guangdong Province, China; ^5^Department of Gastroenterology, The Third Affiliated Hospital of Sun Yat-Sen University, No. 600 Tianhe Road, Guangzhou, 510000 Guangdong Province, China

## Abstract

**Objective:**

This systematic review and meta-analysis aimed to compare the diagnostic performance of transient elastography (TE) and two-dimensional shear wave elastography (2D-SWE) for staging liver fibrosis in patients with chronic viral hepatitis (CVH).

**Methods:**

Pubmed, Embase, Web of Science, and Cochrane Library were searched (-01/08/2021) for studies comparing TE with 2D-SWE in patients with CVH. Other etiologies of chronic liver disease (CLD) and articles not published in SCI journals were excluded. The bivariate random-effects model was used to pool the performance of the TE and 2D-SWE.

**Results:**

Eight articles with a total of 1301 CVH patients were included. The prevalence of significant fibrosis (fibrosis stage ≥ 2), advanced fibrosis (fibrosis stage ≥ 3), and cirrhosis was 50.8%, 44.8%, and 34.7%, respectively. 2D-SWE expressed higher overall accuracy than TE in detecting significant fibrosis (0.93 vs. 0.85, *P* = 0.04). No significant difference among the overall diagnostic accuracy of TE and 2D-SWE in staging advanced fibrosis and cirrhosis was found.

**Conclusion:**

TE and 2D-SWE express good to excellent diagnostic accuracies to stage fibrosis in CVH patients. 2D-SWE compares favorably with TE especially for predicting significant fibrosis.

## 1. Introduction

As the leading cause of liver fibrosis and subsequent hepatocellular carcinoma, chronic viral hepatitis (CVH) infection affects approximately 325 million people worldwide and thus contributing significantly to the global health burden [1]. Liver fibrosis is an important pathological basis of liver cirrhosis in patients with chronic viral hepatitis. Accurate assessment of liver fibrosis degree is of great clinical importance in deciding optimal antiviral treatment time, monitoring dynamic changes of chronic viral hepatitis, and identifying candidates for surveillance for hepatocellular carcinoma [2, 3]. Early-stage liver fibrosis is potentially reversible, but precise diagnoses are often difficult to achieve [4]. Liver biopsy is the gold standard, but it is an invasive examination with potential risks, poor repeatability, and certain limitations, limiting its use in routine clinical practice. A rapid, noninvasive, and straightforward method to identify early-stage liver fibrosis has become increasingly popular.

Transient elastography (TE), two-dimensional shear wave elastography (2D-SWE), and pathological biopsy show great mutual agreement. As the most widely used device based on TE, FibroScan is the World Health Organization recommended diagnosis tool for grading liver fibrosis [5, 6]. 2D-SWE is another well-validated elastography technique using conventional ultrasound diagnostic system, which can quantitatively evaluate the elastic modulus of tissue in a certain selected area [7]. 2D-SWE also displays excellent diagnostic utility for liver fibrosis in chronic hepatitis B (CHB) or chronic hepatitis C (CHC) patients [8, 9].

The severity of liver fibrosis has been known to be a crucial risk factor for hepatocellular carcinoma development. Most patients sequentially develop hepatitis, fibrosis, cirrhosis, and then hepatocellular carcinoma. Given that hepatocellular carcinoma is most often associated with CVH infection (including hepatitis B and C) and toxic exposure [10], staging the degree of fibrosis in CVH is vital for stratification of the risk for hepatocellular carcinoma development, contributing to the management of these patients. Deffieux et al. [11] reported that TE expressed similar diagnostic performance to 2D-SWE in CVH patients. However, a meta-analysis based on the individual data implied that 2D-SWE outperformed TE in CVH patients [12]. Whether 2D-SWE is superior to TE for fibrosis, CVH remains under debate. To determine a better imaging technique for the fibrosis of CVH, we conduct a meta-analysis, including only articles with head-to-head comparison between TE and 2D-SWE.

## 2. Materials and Methods

We performed this systematic review following the PRISMA (Preferred Reporting Items for Systematic Reviews and Meta-Analyses) guideline [13]. Our review protocol was registered at PROSPERO with number CRD42021272672. This study is a meta-analysis of previous research data and ethics statement is not applicable.

### 2.1. Articles Search Strategy

The key words “hepatitis B,” “hepatitis C,” “chronic viral hepatitis,” “liver fibrosis,” “FibroScan,” “transient elastography,” “shear wave elastography,” “Supersonic shear imaging,” “SSI,” or “ShearWave^TM^ elastography” were used to search in Pubmed, Embase, the Web of Science, and the Cochrane Library (-01/10/2021).

### 2.2. Eligibility Criteria

The inclusion criteria are as follows: (1) the accuracies of 2D-SWE and TE for liver fibrosis in patients with hepatitis B virus (HBV) or hepatitis C virus (HCV) were investigated. The paired data of the studies with head-to-head comparison of TE and 2D-SWE was sufficient to construct 2 × 2 table of test performance; (2) the specific liver fibrosis stage was confirmed by biopsy and the (3) the original articles could be retrieved from SCI journals. The exclusion criteria included the following: (1) studies did not assess the accuracies of TE and 2D-SWE; (2) conference abstracts, review, meta-analysis, case report, and other special types of work were not considered; (3) diagnosis of alcoholic liver disease (ALD), nonalcoholic fatty liver disease (NAFLD), autoimmune liver disease, or hepatic carcinoma.

### 2.3. Identification of Liver Fibrosis

Regarding the liver histological assessment, the Metavir, Scheuer, and Ishak scoring system were both included in this research. If the fibrosis stage was assessed with the Metavir or Scheuer system, fibrosis was scored as follows: *F*0, no fibrosis; *F*1, mild/moderate fibrosis; *F* ≥ 2, significant fibrosis; *F* ≥ 3, advanced fibrosis; and *F*4, cirrhosis. According to the Ishak scoring system, fibrosis was scored as follows: *F* 0-1, no/mild fibrosis; *F* ≥ 2, moderate fibrosis; *F* ≥ 3, significant fibrosis; *F* ≥ 4, advanced fibrosis; and *F* ≥ 5, cirrhosis.

### 2.4. Data Collection and Quality Evaluation

At the initial screening stage, two experienced researchers make preliminary selections following the eligibility criteria. Each reviewed the author then extracted the data individually. We then assessed the quality of the included studies with Quality Assessment of Diagnostic Accuracy Studies (QUADAS-2) tool via Review Manager 5.3 (The Cochrane Collaboration). If discrepancies exist, a third research would independently perform proofreading. Discrepancies were further discussed to achieve a high level of agreement if necessary.

### 2.5. Statistical Analysis

Based on the constructed 2 × 2 table with the number of true positives (tp), false positives (fp), false negatives (fn), and true negatives (tn), the summary positive likelihood ratio (LR) and negative LR were acquired following corresponding formulas. For diagnostic accuracy meta-analysis, we adopted a random-effects model (Der Simonian and Laird method). The pooled sensitivity, specificity, summary diagnostic odds ratios (DORs), and the nonthreshold heterogeneity of all the included studies were calculated by Stata (version 16.0) using Midas commands [14]. *I* − squared value > 50% and *P* value < 0.05 were considered suggestive of statistical heterogeneity [15]. We used Metadisc version 1.4 to explore the potential heterogeneity correlated with threshold effect, based on the Spearman correlation coefficient analysis. *P* < 0.05 which indicated significant threshold effects. Publication bias was assessed with Deeks' funnel plots in Stata 16.0. Bivariate random-effects model and hierarchical summary receiver operating characteristic (SROC) analysis were processed using Stata version 16.0. To compare the sensitivity and specificity between different approaches, the *Z* test was performed. The DeLong test was performed to compare ROC curves between TE and 2D-SWE [16]. Statistical significance was assigned as *P* < 0.05.

## 3. Results

### 3.1. Study Characteristics

Figure 1 depicts the study selection process. A total of 6963 potential publications were collected following the search scheme. After deleting duplicates, a total of 4458 publications left. After excluding patent, case report, review, and so forth, 256 articles with full text were downloaded for further screening. By reading the full text, 8 studies [11, 17, 18, 20–24] were ultimately included. Tables 1 and 2 depict both basic and technical characteristics and the technical characteristics of the included studies.  Table 3 depicts the data of diagnostic performance of the studies. The prevalence of significant fibrosis, advanced fibrosis, and cirrhosis was 50.8%, 44.8%, and 34.7%, respectively. A total of 1301 subjects (mean age, 41.5 years; 70.2% male) were included. In addition to 1 (12.5%) retrospective studies, the remaining 7 articles were prospective trials. The details of the QUADAS-2 score are presented in Figure 2. Three (37.5%) publications scored 14 points. Two (25%) studies scored 13 points and 3 (37.5%) studies scored 12 points, respectively.

### 3.2. Diagnosing Significant Fibrosis (F0-1 vs. F2-4)

Eight studies (1301 patients) provided detailed results of head-to-head comparison among TE and 2D-SWE for grading significant fibrosis.  Table 4 summarizes the overall diagnostic performance of TE and 2D-SWE for grading significant fibrosis. The pooled sensitivity and specificity of TE were 0.78 (95% CI, 0.72-0.84) and 0.79 (0.71-0.86), respectively.  Figure 3(a) shows that the summary AUROC of TE was 0.85 (95% CI, 0.82-0.88). The pooled sensitivity and specificity of 2D-SWE were 0.84 (95% CI, 0.78-0.88) and 0.84 (95% CI, 0.77-0.88).  Figure 3(b) shows that the AUROC was 0.90 (95% CI, 0.88-0.93). Compared with TE, 2D-SWE displayed greater sensitivity (0.84 vs. 0.78, *P* < 0.01) and specificity (0.84 vs. 0.79, *P* < 0.01). According to the Delong test, 2D-SWE displays higher accuracy than TE (*Z* = 2.51, *P* = 0.01).

### 3.3. Diagnosing Advanced Fibrosis (F0-2 vs. F3-4)

Six studies (1089 patients) provided detailed results of head-to-head comparison among TE and 2D-SWE for determining advanced fibrosis.  Table 4 summarizes the overall diagnostic performance of TE and 2D-SWE for grading advanced fibrosis. The pooled sensitivity and specificity of TE were 0.85 (95% CI, 0.81-0.89) and 0.88 (95% CI, 0.81-0.93), respectively.  Figure 4(a) shows that the summary AUROC of TE was 0.91 (95% CI, 0.88-0.93). The pooled sensitivity and specificity of 2D-SWE were 0.88 (95% CI, 0.82-0.92) and 0.85 (95% CI, 0.77-0.91).  Figure 4(b) shows that the AUROC was 0.93 (95% CI, 0.90-0.95). The sensitivity of 2D-SWE and TE was similar (0.85 vs. 0.88, *P* = 0.4). 2D-SWE displays similar specificity with TE (0.88 vs. 0.85, *P* = 0.5). According to the Delong test, the overall diagnostic accuracies of TE and 2D-SWE were comparable (*Z* = 1.1, *P* = 0.27).

### 3.4. Diagnosing Cirrhosis (F0-3 vs. F4)

Six studies (1089 patients) provided detailed results of head-to-head comparison among TE and 2D-SWE in detecting cirrhosis.  Table 4 summarizes the overall diagnostic performance of TE and 2D-SWE for grading cirrhosis. The pooled sensitivity and specificity of TE were 0.90 (95% CI, 0.83-0.94) and 0.91 (95% CI, 0.84-0.95).  Figure 5(a) shows that the summary AUROC of TE was 0.95 (95% CI, 0.93-0.97). The pooled sensitivity and specificity of 2D-SWE were 0.95 (95% CI, 0.85-0.99) and 0.91 (95% CI, 0.86-0.95).  Figure 5(b) shows that the AUROC was 0.97 (95% CI, 0.95-0.98).

The sensitivity of 2D-SWE and TE was similar (0.90 vs. 0.95, *P* = 0.19). 2D-SWE displays similar specificity with TE (0.91 vs. 0.91, *P* = 0.87). According to the Delong test, 2D-SWE expressed similar diagnostic accuracy with TE (*Z* = 1.57, *P* = 0.12).

### 3.5. Heterogeneity and Publication Bias

Table 5 summarized the heterogeneity between the included studies. No obvious heterogeneity was observed. The result of Deek's test showed no potential publication bias for TE and 2D-SWE for staging fibrosis.

## 4. Discussion

It is well known that the progression of liver fibrosis can result in increased mortality, mainly due to esophageal-gastric varices bleeding, hepatic encephalopathy, and hepatocellular carcinoma. Chronic infections due to HBV and HCV are responsible for most cases of hepatocellular carcinoma worldwide. Despite promising advances in treatment of hepatocellular carcinoma, ultimately prevention can reduce the burden of viral hepatitis-related hepatocellular carcinoma. Effective monitoring and surveillance for hepatocellular carcinoma must be offered to patients who already have advanced fibrosis or cirrhosis, so that hepatocellular carcinoma is detected at earlier stages, allowing for curative treatments and longer survival. Though liver biopsy remains the gold standard for grading fibrosis, it is not routinely performed due to the invasiveness, sampling error, interobserver variations, and complications of this procedure. Noninvasive tests for evaluation of liver fibrosis mainly include serum biomarkers and measurement of liver stiffness based on elastography. Though serum biomarkers are good reproducibility and high applicability, most of them are nonspecific of the liver and unable to discriminate between intermediate stages of fibrosis [25]. Unlike MR elastography, elastography based on ultrasound machine is less costly, less time-consuming, and widely available, significantly lowering the barriers of clinical application [26]. Growing evidence indicate that TE and 2D-SWE express excellent diagnostic performance for liver fibrosis in CVH.^11-12^ Whether 2D-SWE outperforms TE for fibrosis, CVH remains controversial. Therefore, we conduct this meta-analysis to determine a better technique for patients with CVH.

Our meta-analysis concludes that TE and 2D-SWE show acceptable diagnostic accuracies to stage fibrosis in people with CVH. 2D-SWE outperforms TE in predicting significant fibrosis (AUROCs = 0.90 vs. 0.85, *P* = 0.01). Compared with TE, significantly improved sensitivity (0.84 vs. 0.78, *P* < 0.01) and specificity (0.84 vs. 0.79, *P* < 0.01) was seen for detecting significant fibrosis using 2D-SWE. According to hepatitis B management guidances proposed by the American Association for the Study of Liver Diseases (AASLD), we need to initiate antivirus treatment with elevated HBV DNA levels and histologic evidence of significant fibrosis [27]. Therefore, the advantage of 2D-SWE is evident in the management of HBV-infection, which was similar to an individual patient data based meta-analysis [12]. Our result may also help guide the treatment for patients with chronic hepatitis C. According to the guidelines from the American Association of Liver Diseases, HCV patients without cirrhosis can receive pibrentasvir (120 mg)/glecaprevir (300 mg) for 8 weeks. For cirrhotic patients, they are suitable for velpatasvir (100 mg)/sofosbuvir (400 mg) for 12 weeks [28]. Since 2D-SWE expressed similar diagnostic accuracy with TE in predicting cirrhosis, TE and 2D-SWE were both the ideal candidate for patients with HCV. Nevertheless, this finding seems not generalisable to other etiologies. As indicated by another latest meta-analysis, neither TE nor 2D-SWE met the minimum acceptable performance for detecting significant fibrosis in NAFLD. The respective summary AUROCs of 2D-SWE and TE are 75% and 83% [29]. The difference between CVH and NAFLD may be attributed to the higher prevalence of obesity and hepatic steatosis in NAFLD patients. The diagnostic performance of TE would be substantially affected when patients have obesity, ascites, or steatosis [30]. Steatosis is also one of the confounding factors of 2D-SWE. A latest study based on 1306 patients with liver biopsy found that 2D-SWE might be affected by moderate to severe liver steatosis in diagnosing significant fibrosis [31]. No head-to-head comparison between TE and 2D-SWE was performed in patients with ALD for liver fibrosis. Based on the current evidence, only TE is recommend as a noninvasive tool in patients with chronic harmful alcohol use. Liver stiffness measurement by TE < 8 kPa is recommended to rule-out advanced fibrosis in clinical practice [32]. More prospective and multicenter studies on the diagnostic performance of 2D-SWE are needed to provide robust evidence in patients with ALD.

For discriminating advanced fibrosis and cirrhosis, 2D-SWE displays similar overall diagnostic accuracy with TE (AUROCs = 0.93 vs. 0.91, *P* = 0.27; AUROCs = 0.97 vs. 0.95, *P* = 0.12). The overall diagnostic performance of TE for staging advanced fibrosis and cirrhosis in CVH is similar to a previous meta-analysis based on 4386 CHB patients, with summary AUROCs of 0.91 and 0.93, respectively [33]. A recent meta-analysis based on 5126 CHB patients shows that the summary AUROC values of 2D-SWE for advanced fibrosis and cirrhosis were 0.93 and 0.94 [34]. The summary AUROCs of TE or 2D-SWE in our results are higher than theirs. Since we only include studies with head-to-head comparison of TE and 2D-SWE, numerous articles were excluded. As a result, the outcome of our meta-analysis is likely to overestimate accuracy, given the small sample sizes examined (*n* = 1089). TE and 2D-SWE also displays similar diagnostic accuracy for staging advanced fibrosis and cirrhosis in patients with biopsy-proven NAFLD [35, 36].

Except for the overall diagnostic accuracy, we also investigated the rates of reliable liver stiffness measurements of the two examinations in patients with CVH. The technical failure rate of 2D-SWE was below or equal to that of TE (Table 2), indicating that 2D-SWE is a preferable technique providing more reliable measurement. Moreover, compared with TE, 2D-SWE allows an easier access to the certain selected area [37], facilitating the monitoring of the variation of blood flow [38, 39].

With further study, 2D-SWE demonstrates enormous potential for prognosis prediction in patients with CVH. Wu et al. [40] proposed that liver stiffness measured with 2D-SWE is predictive of liver-related events in patients with HBV. 2D-SWE has recently exhibits great potential for redoing the burden of viral hepatitis-related hepatocellular carcinoma. A multivariable model based on age, platelets, and the liver stiffness measured by 2D-SWE can accurately predicts hepatocellular carcinoma in CHB during five-year follow-up, with an AUROC of 0.89 [41]. Another study from Korea implies that liver stiffness value measured by 2D-SWE was a significant predictive factor for overall survival after radiofrequency ablation for hepatocellular carcinoma [42]. Liver stiffness measured by 2D-SWE could also stratify the risk of symptomatic post-hepatectomy liver failure in Child-Turcotte-Pugh grade A patients, regardless of the extent of hepatectomy [43]. This demonstrates that 2D-SWE is a better choice to stage fibrosis.

The strengths of this meta-analysis were summarized as follows: studies comparing the diagnostic performance within the same patient provide a more valid way of comparing different tests. Hence, our meta-analysis is persuasive as we only included studies with head-to-head comparisons between TE and 2D-SWE. Moreover, no substantial heterogeneity was observed. The corresponding results are more convincing and reliable. However, limitations still exist. First, we did not evaluate the potential confounding factors such as obesity, tissue inflammation, and the quantification of viral activity, which may affect the diagnostic accuracies [44]. Although the diagnostic performance of 2D-SWE may not be affected by BMI and liver function indexes [45], TE tends to be affected by inflammation and cholestasis [46] and thus affecting our judgments. Additionally, because of the limited studies in patients with HCV and no substantial heterogeneity observed in the meta-analysis, we did not separately investigate the performance of elastography among patients with HBV or HCV.

## 5. Conclusion

Collective, TE and 2D-SWE display good to excellent accuracies in staging fibrosis in patients with HBV or HCV. 2D-SWE compares favorably with TE especially for predicting significant fibrosis.

## Figures and Tables

**Figure 1:** Flow diagram of the study selection. 150 × 160 mm (300 × 300 DPI).

**Figure 2:** Summary of methodological quality of 8 studies according to Quality Assessment of Diagnostic Studies-2 (QUADAS-2) tool. (a) Overall and (b) study-level of bias. 150 × 160 mm (300 × 300 DPI).

**Figure 3:** The SROC curves of TE and 2D-SWE showing performance in staging fibrosis stage *F* ≥ 2. (a) SROC plot of TE for fibrosis stage *F* ≥ 2. (b) SROC plot of 2D-SWE for fibrosis stage F ≥ 2. 2D-SWE: two-dimensional shear wave elastography; SROC: summary receiver operating characteristic; TE: transient elastography. 150 × 75 mm (300 × 300 DPI).

**Figure 4:** The SROC curves of TE and 2D-SWE showing performance in staging fibrosis stage *F* ≥ 3. (a) SROC plot of TE for fibrosis stage *F* ≥ 3. (b) SROC plot of 2D-SWE for fibrosis stage *F* ≥ 3. 2D-SWE: two-dimensional shear wave elastography; SROC: summary receiver operating characteristic; TE: transient elastography. 150 × 75 mm (300 × 300 DPI).

**Figure 5:** The SROC curves of TE and 2D-SWE showing performance in staging cirrhosis. (a) SROC plot of TE for fibrosis stage *F* = 4. (b) SROC plot of 2D-SWE for fibrosis stage *F* = 4. 2D-SWE: two-dimensional shear wave elastography; SROC: summary receiver operating characteristic; TE: transient elastography. 150 × 75 mm (300 × 300 DPI).

**Table 1:** basic characteristics of the included studies.

Id	Region	Design	Center	Study time	Subject	Mean age	Male (%)	BMI (kg/m^2^)	ALT (U/L)	Etiology	Scoring system	Length of biopsy samples	QUADAS scores
Leung [17]	China	Prospective	Single center	2011-2012	226	48.8	65	24.2 (21.6-27.3)†	69 (37.5-105)†	HBV	Metavir	≥15 mm	12
Yao [22]	China	Prospective	Single center	2013-2015	54	36.7	76	23.9 (21.9-25)†	50.4 (28.8-129.2)†	HBV	Ishak	≥20 mm	14
Zeng [18]	China	Prospective	Single center	2013-2015	257	36.7	77.4	21.7 (19.7-23.9)†	42 (28.3-67.8)†	HBV	Metavir	≥15 mm	13
Ferraioli [21]	Italy	Retrospective	Single center	2010-2012	121	44.8	71.9	25.4 (17.1-39)§	75 (40-126)†	HCV	Metavir	≥10 mm	14
Deffieux [11]	France	Prospective	Single center	2011-2012	70	46.8	79	24.1 (16.7-35.9)§	81.3 (15-260)§	HBV (*n* = 24)HCV (*n* = 46)	Metavir	≥9 mm	14
Xia 2019	China	Prospective	Single center	2017	158	38.55	60.1	NA	NA	HBV	Scheuer	≥15 mm	12
Paul [23]	India	Prospective	Single center	2012-2014	240	32.6	73.3	22.3 ± 4.1	71.7 ± 89.0	HBV (*n* = 172) HCV (*n* = 68)	Metavir	≥10 mm	12
Osman [24]	Egypt	Prospective	Single center	2019	180	51.07	65	NA	NA	HBV (*n* = 32) HCV (*n* = 148)	Metavir	NA	13

^∗^Mean ± SD. †Median (interquartile range). §Median (range). BMI: body mass index; NA: not available; QUADAS: quality assessment of studies of diagnostic accuracy studies; TE: transient elastography.

**Table 2:** Technical characteristics of the included studies.

Id	TE				2D-SWE				
	No. of reader	Experience of operator	Probe	Technical failure rate	No. of reader	Experience of operator	Probe	Diameter of ROI	Technical failure rate
Leung [17]	1	More than 5 years	NA	10.4% (47/454)	1	NA	SC6-1	3-4 cm	1.1% (5/454)
Yao [22]	1	At least 100 TE procedures	M	0	1	NA	SC6-1	2 cm	0
Zeng [18]	2	At least 100 TE procedures	M	3.1% (8/257)	2	More than 6 months	SC6-1	2 cm	0.8% (2/257)
Ferraioli [21]	1	At least 50 TE procedures	NA	2.5% (3/121)	2	NA	SC6-1	2 cm	1.7% (2/121)
Deffieux [11]	1	More than 7 years	NA	5.3% (6/114)	2	NA	SC6-1	3 cm	1.7% (2/120)
Xia 2019 [19]	NA	NA	M or L	NA	2	NA	L5-1	NA	NA
Paul [23]	NA	NA	M or XL	2.1% (5/240)	NA	NA	SC6-1	1-1.5 cm	1.3% (3/240)
Osman [24]	1	NA	NA	14.0% (30/210)	1	NA	NA	NA	5.7% (12/210)

2D-SWE: two-dimensional shear wave elastography; NA: not available; ROI: region of interest; QUADAS: quality assessment of studies of diagnostic accuracy studies; TE: transient elastography.

**Table 3:** Data of diagnostic performance of the studies included in the meta-analysis.

Study id	Staging fibrosis stage *F* ≥ 2						Staging fibrosis stage *F* ≥ 3						Staging fibrosis stage *F* = 4					
	Sensitivity		Specificity		AUROC		Sensitivity		Specificity		AUROC		Sensitivity		Specificity		AUROC	
	TE	2D-SWE	TE	2D-SWE	TE	2D-SWE	TE	2D-SWE	TE	2D-SWE	TE	2D-SWE	TE	2D-SWE	TE	2D-SWE	TE	2D-SWE
Leung [17]	0.78	0.85	0.81	0.92	0.78	0.88	0.81	0.9	0.92	0.9	0.83	0.93	0.92	0.97	0.92	0.92	0.92	0.98
Yao [22]	0.59	0.78	0.67	0.78	0.71	0.79	NA	NA	NA	NA	NA	NA	NA	NA	NA	NA	NA	NA
Zeng [18]	0.79	0.89	0.81	0.76	0.85	0.88	0.86	0.90	0.78	0.77	0.88	0.92	0.94	0.94	0.83	0.87	0.91	0.93
Ferraioli [21]	0.70	0.90	0.90	0.88	0.84	0.92	0.89	0.97	0.89	0.95	0.96	0.98	0.92	0.88	0.97	0.97	0.96	0.98
Deffieux [11]	0.84	0.87	0.82	0.76	0.89	0.85	0.81	0.86	0.83	0.74	0.83	0.82	0.78	1.00	0.86	0.79	0.87	0.90
Xia 2019 [19]	0.80	0.76	0.56	0.91	0.75	0.94	0.94	1.00	0.86	0.91	0.87	0.97	0.86	0.89	0.86	0.96	0.91	0.97
Paul [23]	0.75	0.67	0.78	0.70	0.84	0.76	0.82	0.81	0.83	0.78	0.90	0.90	0.83	0.83	0.97	0.91	0.97	0.93
Osman [24]	0.91	0.89	0.89	0.85	0.95	0.93	0.93	0.90	0.97	0.95	0.90	0.98	0.96	1.00	0.97	0.91	0.97	0.93

2D-SWE: two-dimensional shear wave elastography; AUROC: area under summary receiver operating characteristic; NA: not available; TE: transient elastography.

**Table 4:** Meta-analysis of studies with head-to-head comparison of TE and 2D-SWE in staging fibrosis.

Methods	No. of studies (no. of patients)	Cutoff values range	Sensitivity (95% CI)	Specificity (95% CI)	PLR (95% CI)	NLR (95% CI)	AUROC(95% CI)	DOR (95% CI)
Staging fibrosis stage *F* ≥ 2								
TE	8 (1301)	6.1-11.8	0.78 (0.72-0.84)	0.79 (0.71-0.86)	3.71 (2.43-5.67)	0.28 (0.21-0.38)	0.85 (0.82-0.88)	14.12 (7.88-25.31)
2D-SWE	8 (1301)	6-9.58	0.84 (0.78-0.88)	0.84 (0.77-0.88)	4.87 (3.22-7.36)	0.2 (0.13-0.32)	0.90 (0.88-0.93)	25.19 (11.47-55.32)
Staging fibrosis stage *F* ≥ 3								
TE	6 (1089)	8-8.6	0.85 (0.81-0.89)	0.88 (0.81-0.93)	7.05 (4.04-12.32)	0.17 (0.12-0.24)	0.91 (0.88-0.93)	44.23 (20.5-95.43)
2D-SWE	6 (1089)	7-9.1	0.88 (0.82-0.92)	0.85 (0.77-0.91)	6.19 (371-10.30)	0.14 (0.08-0.23)	0.93 (0.90-0.95)	50.24 (21.09-119.69)
Staging fibrosis stage *F* = 4								
TE	6 (1089)	11.2-14.6	0.90 (0.83-0.94)	0.91 (0.84-0.95)	10.7 (5.46-20.99)	0.11 (0.05-0.24)	0.95 (0.93-0.97)	110.24 (40.75-298.24)
2D-SWE	6 (1089)	9.7-11.3	0.95 (0.85-0.99)	0.91 (0.86-0.95)	9.34 (5.91-14.76)	0.07 (0.02-0.27)	0.97 (0.95-0.98)	155.43 (63-383.43)

2D-SWE: two-dimensional shear wave elastography; AUROC: area under summary receiver operating characteristic; CI: confidence interval; DOR: diagnostic odds ratio; NLR: negative likelihood ratio; PLR: positive likelihood ratio; TE: transient elastography.

**Table 5:** Heterogeneity of all the included studies.

Staging fibrosis	Threshold heterogeneity		Nonthreshold heterogeneity	
	*r*_*s*_	*P* value	*I* ^2^	*P* value
TE				
Staging fibrosis stage ≥ 2	-0.12	0.78	0.54	0.06
Staging fibrosis stage ≥ 3	-0.26	0.62	0.51	0.07
Staging cirrhosis	-0.37	0.47	0	0.25
2D-SWE				
Staging fibrosis stage ≥ 2	-0.1	0.82	0.56	0.05
Staging fibrosis stage ≥ 3	-0.66	0.16	0	0.24
Staging cirrhosis	-0.14	0.79	0.47	0.08

2D-SWE: two-dimensional shear wave elastography; TE: transient elastography.

## Data Availability

The datasets used and/or analyzed during the current study are available from the corresponding author on reasonable request.

## Abbreviations

AASLD: American Association for the Study of Liver Diseases
AUROC: Area under the receiver operating characteristic curve
CHB: Chronic hepatitis B
CHC: Chronic hepatitis C
CVH: Chronic viral hepatitis
DOR: Diagnostic odds ratio
HBV: Hepatitis B virus
HCV: Hepatitis C virus
LR: Likelihood ratio
NAFLD: Nonalcoholic fatty liver disease
NPV: Negative predictive value
PPV: Positive predictive value
QUADAS: Quality assessment of diagnostic accuracy studies
ROC: Receiver operating characteristic
ROI: Region of interest
2D-SWE: Two-dimensional shear wave elastography
TE: Transient elastography.
